The article "Multistage Optimization Using a Modified Gaussian Mixture Model in Sperm Motility Tracking" was published in 2021. Journal: Comput Math Methods Med.

# Multistage Optimization Using a Modified Gaussian Mixture Model in Sperm Motility Tracking

**DOI:** 10.1155/2021/6953593

**Published:** 2021-08-29

**Authors:** Mohammed Alameri, Khairunnisa Hasikin, Nahrizul Adib Kadri, Nashrul Fazli Mohd Nasir, Prabu Mohandas, Jerline Sheeba Anni, Muhammad Mokhzaini Azizan

**Affiliations:** ^1^Department of Biomedical Engineering, Faculty of Engineering, Universiti Malaya, Lembah Pantai, 50603 Kuala Lumpur, Malaysia; ^2^Biomedical Electronic Engineering Program, Faculty of Electronic Engineering Technology, Universiti Malaysia Perlis, Pauh Putra Campus, 02600 Arau, Perlis, Malaysia; ^3^Sport Engineering Research Centre (SERC), Universiti Malaysia Perlis, Pauh Putra Campus, 02600 Arau, Perlis, Malaysia; ^4^Department of Computer Science and Engineering, National Institute of Technology Calicut, Kerala, India; ^5^Department of Computer Science and Engineering, MEA Engineering College, Kerala, India; ^6^Department of Electrical and Electronic Engineering, Faculty of Engineering and Built Environment, Universiti Sains Islam Malaysia, Bandar Baru Nilai, 71800 Nilai, Negeri Sembilan, Malaysia

## Abstract

Infertility is a condition whereby pregnancy does not occur despite having unprotected sexual intercourse for at least one year. The main reason could originate from either the male or the female, and sometimes, both contribute to the fertility disorder. For the male, sperm disorder was found to be the most common reason for infertility. In this paper, we proposed male infertility analysis based on automated sperm motility tracking. The proposed method worked in multistages, where the first stage focused on the sperm detection process using an improved Gaussian Mixture Model. A new optimization protocol was proposed to accurately detect the motile sperms prior to the sperm tracking process. Since the optimization protocol was imposed in the proposed system, the sperm tracking and velocity estimation processes are improved. The proposed method attained the highest average accuracy, sensitivity, and specificity of 92.3%, 96.3%, and 72.4%, respectively, when tested on 10 different samples. Our proposed method depicted better sperm detection quality when qualitatively observed as compared to other state-of-the-art techniques.

## 1. Introduction

Infertility is a medical condition that is represented by the failure of the reproduction system to produce children. Several factors lead to this condition such as genetic disorder, HIV, diabetes, cancer, or overexposure to certain environmental factors [1]. Globally, there are approximately between 48.5 and 52 million reported cases with infertility cases which is estimated to be around 15% of the total couples around the world [2]. In Malaysia, the Government Department of Statistics reported a fertility rate drop from 4.9 to 1.8 babies per woman between 1970 and 2018. The infertility issue originates from either the man or the woman or in some cases; both couples contribute to the problems [3, 4]. In most male infertility cases, sperm disorder is considered to be the most common cause of the infertility [4]. Males alone are responsible for 20–30% of the infertility disorder, and they contribute around 50% of the overall causes [5].

The article "Multistage Optimization Using a Modified Gaussian Mixture Model in Sperm Motility Tracking" was published in 2021. Journal: Comput Math Methods Med.

There are several ways to diagnose the infertility issue among men such as constant measurement of blood and hormone levels, physical exams, and pH level [6]. However, these approaches rely on manual assessments which are prone to human error, costly, and time-consuming. Another approach is through semen analysis which relies on examining and evaluating the properties of the sperm, and it has been widely explored. Generally, there are three ways to analyze the sperm, namely, (1) sperm count—which concerns about the concentration of the sperms within a sample, (2) sperm morphology—which depends on examining the shape and the size of the sperm's structure, and (3) sperm motility—which estimates the velocity of the sperm. These three properties provide clues to detect infertility and can indicate the overall quality of the sperm [7, 8]. The World Health Organization (WHO) has established a standard to identify the normal and the abnormal sperm based on these three criteria as tabulated in Table 1 [9].

Sperm analysis is a powerful tool to examine the fertility disorder, and Table 1 tabulates the cut-off values for the sperm parameters. In other words, if the obtained value for the analyzed case is less than the cut-off, then, the case is considered abnormal. Approximately two out of six men in the world are having fertility issues, and around 30% of them encounter problems associated with sperm quality. There are several ways to investigate the sperm properties such as sperms' DNA fragmentation and sperm chromatin structure assay. However, these methods are time-consuming and costly and need to be handled manually. Therefore, new methods have been introduced based on computer vision which includes the modification of image processing techniques to analyze sperm's properties. The use of computer vision in the sperm analysis has provided several advantages such as the following: (i) it provides a rapid diagnosis, (ii) it can be modified, (iii) it does not require other chemical condition, and (iv) it is less prone to human error.

This paper is divided into 5 main sections, of which each of them describes the work undertaken for the completion of this research. In Introduction, this paper explores the general understanding of infertility from a global perspective, especially on worldly accepted WHO standard. The cause behind infertility is also looked into, in order to understand the background as well the available diagnostic processes related to the issue. In Research Background, gap analysis was performed through comparisons between currently available methodologies and techniques. Critical discussions on the latest documents on sperm tracking methodologies with their respective ups and downsides are discussed. Findings inside this section provided the motivation behind this manuscript and the way modified Gaussian Mixture Modelling suit the founded gap. Within Methodology, this manuscript discussed the modified Gaussian Mixture Modelling (GMM) which includes the introduction of optimization of sperm detection and the subsequent sperm motility tracking which now uses the input of the optimized detection techniques. Based on the work done in this section, the results are discussed on three main parameters that are accuracy (*A*), sensitivity (Sn), and specificity (Sp). In Results, the outcome of the proposed modified GMM is benchmarked with a few known, similar techniques to evaluate its performance. Several concluding remarks were performed in Conclusion, where the performance of the proposed algorithm is described to highlight strength and challenges of the work.

The article "Multistage Optimization Using a Modified Gaussian Mixture Model in Sperm Motility Tracking" was published in 2021. Journal: Comput Math Methods Med.

## 2. Research Background

Although sperm count and morphology can give some indications about the statue of the sperms, they are considered nonreliable to draw a decisive conclusion on the fertility on the male in comparison to sperm motility analysis [10]. Since the main concern in fertility analysis is the first sperm that reaches the fallopian tube and fertilizes the egg, therefore, studying the sperm's velocity properties could provide more accurate results. According to the WHO, sperm's motility can be categorized in three terms: (i) fast progressive (FP) which means the sperm motility is with velocity ≥ 25 *μ*m/s, (ii) slow progressive (SP) which means the sperm motility is with velocity < 25 *μ*m/s, and (iii) immotile which means the sperm does not move at all [4, 9, 11].

There are multiple ways to estimate the velocity of the sperm, which are either through manual visual observation or through using computerised image processing tools. The examples of the manual approaches are photoelectric and multiple exposure phonograph (MEP) [4, 12]. Through manual visual observation, sperm velocity estimation is relatively slow, insufficient, and less accurate. On the other hand, semen analysis with image processing techniques uses algorithms of the computer visions to estimate the sperm's motility features which are widely acceptable, reliable, fast, and robust [13]. The capability of image processing and computer vision can be seen in various medical field applications [14–18].

The article "Multistage Optimization Using a Modified Gaussian Mixture Model in Sperm Motility Tracking" was published in 2021. Journal: Comput Math Methods Med.

Computer-Aided Sperm Analysis (CASA) was the first method and was introduced in 1985. This method is capable to estimate the total number of sperms, detects the sperm's morphological features, and estimates the velocity of the sperm. The sperm analysis results may vary among different CASA instruments. It is highly dependent on the sperm concentration where high concentration of semen samples may cause motile sperms to be hardly detected. Despite that, this method fails to detect multiple sperms at the same time. Furthermore, it requires big samples for each experiment, and it is not capable of detecting the loss or reborn sperms [19]. The CASA instrument settings should be standardized to ensure the results are comparable where the error trapping rate and the loss trapping rate should be as low as possible.

Joint Probability Data Association Filter (JPDAF) was adapted to track and measure the velocity of hundreds of sperms simultaneously. JPDAF is a mathematical and statistical approach that works based on an approach Global Nearest Neighbour (GNN) which tracks an object by minimizing within distance variable and maximizing the between distance variables. This feature eliminates sperm's collision conditions that intervene the results, and it measures the proximity of close sperms. However, this method has high computational complexity, and its process termination is slower [20–22].

Another modified approach in sperm tracking is the Hybrid Generative-Discriminative Tracker (HGDT). Hybrid Generative system is for object detection, and Discriminative Tracker is for updating the centroid of each sperm for all frames for velocity estimation. This method has features of adaptive learning from frame to another, which enhances the detection and tracking procedure. The main drawback of HGDT that it works properly with single tracker rather than multiple sperm tracking [23, 24].

A recent paper was published earlier this year in which deep learning in sperm detection and tracking was used. A modified method called Channel and Spatial Resolution together with Discriminative Correlation Filter (CSR-DCF) was implemented. It begins with detection in which the RetinaNet method, a deep neural convolutional network approach, was used. This method extracts the main features of the sperm by feeding the Convolutional Neural Network. According to these features, it detects the rest of the sperms for the whole frames. This method requires a higher computational model and large training data set, which makes it difficult to implement and has slow execution time [25].

The article "Multistage Optimization Using a Modified Gaussian Mixture Model in Sperm Motility Tracking" was published in 2021. Journal: Comput Math Methods Med.

Kheirkhah et al. [26] suggested a method for sperm detection and tracking that is based on Adaptive Distance Tracking (ADT). In this method, the sperm is located by detecting its centroid, and then, its coordinates are determined in each frame. Adaptive Window Average Speed (AWAS) is modified to enhance the accuracy of sperm allocation from frame to another. However, this method works poorly in a highly dense solution or when there are many sperms accumulated in a close region.

Another sperm tracking method was suggested by [27] called Differential Area Trajectory (DAT). In this method, the sperms' location is detected collectively, and at the same time, the footprint is constructed. DAT retains the final results as a velocity function with respect to time in order to estimate the velocity of the sperms. Although this method has a low computational complexity and it is easy to implement, it does not detect the dead and reborn sperms and it does not require a testing data (initial frames) which makes the results less accurate.  Table 2 summarizes the previous techniques that have been used in tracking the motile sperms. From the summary presented in this table, we can highlight few research gaps from the existing literatures:

1. The updating mechanisms to consider newly emerging sperms reenter the field of views are disregarded in sperm's velocity estimation. Thus, the classification between normal and abnormality of the sperm motility is inaccurate
2. The efficiency of sperm motility analysis is often decreased in high density medium where the existing system fails to detect multiple sperms
3. Due to this, manual semen analyses are still being used. However, manual analysis has been challenging due to inconsistency of the semen sample. Reproducibility of the analysis is difficult to be achieved which will lead to misclassification

Therefore, in this paper, an automated multistage tracking system is proposed using sperm motility properties. The automated tracking comprises two stages of sperms' head detection and sperm tracking processes. A new modified Gaussian Mixture Model with an automated optimization protocol was proposed to detect multiple sperms head in image frames extracted from sperm motility video. Then, the output from stage 1 will then be utilized to accurately track the motile sperms and eventually determine their velocity.

The main motivation behind this method is to enhance the quality of sperm analysis by providing high accurate and reliable results. The main technical contributions and novelty of this work are listed below:

1. A modified and optimized GMM function for sperm's head recognition is proposed. With the optimization of determining background threshold, more accurate sperm features can be localized. The proposed modified GMM will be able to localize the sperm's features to be tracked in the second stage of the proposed system
2. Multisperm tracking uses similarity and Euclidean distance methods. The detection of the motile sperms will be updated automatically including the new sperms reentering the field of view. This will ensure accurate sperm's velocity can be determined and calculated
3. Provide overall sperm analysis system with less computational and mathematical complexity. The proposed modified GMM has provided an improved sperm features that will generate automated threshold to localize the region of interest (i.e., sperm morphology)

The article "Multistage Optimization Using a Modified Gaussian Mixture Model in Sperm Motility Tracking" was published in 2021. Journal: Comput Math Methods Med.

## 3. Methodology

In this paper, we developed the new algorithm based on the available VISEM Dataset [32] where the collected data were used to investigate male reproductive function. The sperm motility videos were recorded and examined under a 400 times magnification using an Olympus CX31 microscope. The sample was placed on a heated microscope stage (37°C), and the videos were captured by a microscope-mounted camera and saved as AVI file. The dataset contains motility videos from 85 male participants aged 18 years or older. Summary of the dataset specification is tabulated in Table 3.

The overall algorithm for multistage automated sperm motility tracking is presented in Figure 1. The proposed algorithm consists of two stages where the first stage focuses on the preprocessing task where debris are removed from the original frame. In order to accurately detect the moving sperms, unwanted debris are eliminated since beginning. This approach will help improving computational efficiency of the algorithm in tracing the moving sperms (which will be conducted on the second stage). Then, the cleaned image frame was fed into stage 2 where the center coordinates of the sperms' head were detected. These coordinates were then used for sperm tracking in the consecutive frames. The velocity of the sperm was calculated based on the successful tracked sperm, and thus, classification of normal and abnormal was made according to the recorded average velocity of the motile sperms.

### 3.1. Stage 1: Optimization of Sperm Detection

This stage started with the sperm detection process with the aim to distinguish object of interest (i.e., the sperm) from the background. In addition, the image frames were cleaned by implementing morphological opening and closing operation to remove dead cells or debris in each image frame. Then, a modified Gaussian Mixture Model (GMM) with a new optimization of Gaussian density function is implemented to detect the sperms and separate them from the background. This technique is clustering-based method that assigns each object to a certain class using the mathematical probability of Gaussian density function, (*Ɲ*(*x* | *μ*, *Σ*) to segment the objects of interest from the background as shown in

(1) $$\begin{array}{c} Ɲ\left(x\;|\;\mu ,\Sigma \right)=\frac{1}{{\left(2\pi \right)}^{D/2}{\left|\Sigma \right|}^{1/2}\;}\exp\left(-\frac{1}{2}{\left(x-\mu \right)}^{T}\Sigma^{-1}\left(x-\mu \right)\right), \end{array}$$

where *x* is the pixel intensity value, *μ* is the mean, *Σ* is the covariance matrices, and *D* is the dimension of the matrix.

The article "Multistage Optimization Using a Modified Gaussian Mixture Model in Sperm Motility Tracking" was published in 2021. Journal: Comput Math Methods Med.

The pseudocode of the modified GMM is shown in Figure 2. During this stage, all objects are clustered into two different classes, and every class has a different mean *μ* to estimate its center, covariance *Σ* that indicates its length, and weight probability *π* that describe the how large or small is the class. If the Gaussian density function (*Ɲ*(*x* | *μ*, *Σ*) is bigger than the set threshold, the pixel is considered the object whereas if the (*Ɲ*(*x* | *μ*, *Σ*) is smaller than the predetermined background threshold (BG_T_), the pixel is considered as the background. To ensure accurate and robust detection of the sperm, the set threshold was automatically generated based on the proposed optimization algorithm as shown in Figure 3. The BG_T_ is automatically generated based on the sperm sample. The Gaussian density function is calculated, and the process is repeated to attain the highest detected motile sperms.

To obtain the best value of BG_T_, we used the number of detected sperm as the main parameter to check the accuracy of the sperm detection. Since each sperm motility video is recorded in the same environment for each sample, we only computed the optimization procedure on the first frame of every acquired video. This process will ensure efficient parameter optimization and thus ensuring accurate detection. Therefore, for the highest number of detected sperm attained, the BG_T_, the value is chosen as the best value. The optimized sperm detected video based on the automated computation of *BG_T_* is produced by conducting the proposed optimization technique as shown in Figure 3. The BG_T_ values were set to have ranged from 10% to 100%; therefore, the loop of *i* ≥ 9 was applied to ensure automated generation of the threshold values.

The resulted images from GMM are not clear enough to do further analysis. The reason is that there are a lot of dead cell and derbies that were mixed or surrounded the edges of the sperm. This will lead to misinterpretation on the results and inaccurate velocity measurement. Therefore, morphological process of open and close operations was implemented to reduce the unwanted noise. This technique is based on either dilating or contracting the shape of the object in the background. In this study, image opening and image closing were applied simultaneously to get a clearer image frame. The size of added or removed pixels is represented by the size of the kernel or structural element (SE). Equations (2) and (3) demonstrate the mathematical expression of the image opening and closing, respectively.

(2) $$\begin{array}{c} A\circ B=\left(A⊖B\right)⊕B, \end{array}$$

(3) $$\begin{array}{c} A\circ B=\left(A⊕B\right)⊖B. \end{array}$$

where *A* is the binary image (results of the modified GMM) and *B* is *SE* element.

The article "Multistage Optimization Using a Modified Gaussian Mixture Model in Sperm Motility Tracking" was published in 2021. Journal: Comput Math Methods Med.

### 3.2. Stage 2: Sperm Motility Tracking

Once the optimized detected sperms were found in stage 1, the detection and tracking processes were continued during which the centers of the sperms' heads were identified. Objects that are elliptical and have area of 150 pixel^2^ were considered the object of interest (i.e., sperm). Objects that are less than 150 pixel^2^ are considered debris and were eliminated from the tracking process. The elliptical area is calculated using

(4) $$\begin{array}{c} A_{\text{elliptical}}=\pi *\text{major axes}*\text{minor axes}. \end{array}$$

The coordinates of the sperms' head were recorded for every 10^th^ frame of the sperm motility video. The mathematical procedure of the Mass of the Central Momentum of object was implemented to detect the centers of the sperms' heads. This method is capable of working on multiobject or sperm detection in the same frame. Using the Mass of the Central Momentum technique, the coordinates of the center of the sperms' head are calculated using

(5) $$\begin{array}{c} x_{c}=\frac{n_{1,0}}{n_{0,0}}, \end{array}$$

(6) $$\begin{array}{c} y_{c}=\frac{n_{0,1}}{n_{0,0}}, \end{array}$$

(7) $$\begin{array}{c} n_{1,0}=\iint_{-\infty }^{\infty }dxdyxb\left(x,y\right), \end{array}$$

(8) $$\begin{array}{c} n_{0,1}=\iint_{-\infty }^{\infty }dxdyyb\left(x,y\right), \end{array}$$

where the coordinate of the sperm's head center is donated as (*x*_*c*_, *y*_*c*_), *n*_0,0_ is the zero-order moment that describes the area of the object, and *n*_1,0_ and *n*_0,1_ are specified in Equations (6) and (7), respectively. *b*(*x*, *y*) is the binary image that resulted from stage 1.

This stage is aimed at finding the sperm in the previous frame that is closest and most similar to the sperm in the current frame. There are two assumptions that we made in this stage: (i) the distance between two sperms (i.e. sperms in current frame and previous frame) must not exceed the distance threshold of 125 pixels to be considered the same motile sperm, and (ii) the shape of the sperms' heads and their deformity of the elliptical must not change much in each frame. The threshold of 125 pixels was set based on observation and simulation test on all samples. In addition, the threshold was set by considering the size ratio between sperm's head and tail. Thus, by observing the behaviour of the sperm's movements in all samples, we concluded that the threshold of 125 pixels is acceptable to be used. The closeness of the sperm was defined by having a minimum Euclidean distance between centers of two sperms of *S*_*c*_ (i.e. sperm in the current frame) and *S*_*p*_ (sperm in the previous frame) given by

(9) $$\begin{array}{c} d\left(S_{c},S_{p}\right)=\sqrt{\overset{2}{\underset{i=1}{\sum }}{\left(x_{c}-x_{p}\right)}^{2}+{\left(y_{c}-y_{p}\right)}^{2}\;}\leq t_{dis}. \end{array}$$

Therefore, we measured the ratio of the sperm's head area from the current (for example, frame-20^th^) and the previous frames (for example, frame 10^th^). The ratio should not exceed the threshold which was defined as the positive differences between the area sizes in the current and the previous frames. Equation (10) denotes the mathematical definition of the procedure for tracking process.

(10) $$\begin{array}{c} \text{Similarity}=\left\{\begin{array}{c} 1,\;\text{if }{S_{Z}}_{p}>{S_{Z}}_{c}\text{ and }\frac{{S_{Z}}_{p}}{{S_{Z}}_{c}}\leq t_{\text{size}}\text{ or }{S_{Z}}_{p}<{S_{Z}}_{c}\text{ and }\frac{{S_{Z}}_{c}}{{S_{Z}}_{p}}\leq t_{\text{size}},\\ 0, \end{array}\right.\; \end{array}$$

where *S*_*Z*__*p*_ the area of the sperm in the previous frame and *S*_*Z*__*c*_ is the area of the sperm in the current frame. The results of this equation were automatically updated and stored in a matrix. *t*_size_ is the threshold size that is set to 1.2 in this study with the assumption that the object's size is not expected to change significantly between antecedent and subsequent frames. The threshold was set based on the simulation that was done on 10 different semen samples.

The article "Multistage Optimization Using a Modified Gaussian Mixture Model in Sperm Motility Tracking" was published in 2021. Journal: Comput Math Methods Med.

Based on two conditions as mentioned above, sperms in the current frame were matched with their corresponding frame from the previous frame. If the Euclidean distance and size ratio between sperm in the current and previous frames were less than or equal to the predetermined thresholds, sperm in the previous frame was matched to its corresponding sperm with the sperm in the current frame.

If either closeness or similarity of the object was not achieved, the object was considered the sperm that swims out from the frame. The sperm tracker was reinitialized where the nonmatching sperm was removed from the tracker. If the sperm was successfully matched with its corresponding sperm, the process was repeated until all sperms in the frame were processed. This process was continuously conducted until all image sequence frames were analyzed. Since SE was implemented in the image optimization, the selection of SE does not directly affect the tracking and the detection process. However, the SE was used for morphological operation to improve the clarity of the image and further amplify the sperm's head size, thus indirectly influencing the detection process.

After obtaining the coordinate of the sperms, the sperm's velocity can be measured according to Equation (11). In addition, the unit of the velocity was converted from pixel/second to *μ*m/s (1 pixel = 0.0002 meter) to meet the standard that was stated by the WHO. The centroid was detected once over ten frames so that the variation of the centroid will be large enough for detection to make the system less computational-complex and to increase the processing speed.

(11) $$\begin{array}{c} \text{Velocity}=\frac{\sqrt{{\left(x_{c}-x_{p}\right)}^{2}+{\left(y_{c}-y_{p}\right)}^{2}}}{\text{frame rates}}. \end{array}$$

The frame rate depends on the properties of the video, and its unit is frame per second.

The final velocity result is the average velocity of each sperm in the whole video. The results of sperm's velocity in each detection were stored in a matrix. Then, at the end of the video, the average was obtaining by dividing the summed velocity values in all frames by the number of the frames. This gave the system the feature of detecting the sperms the exited and entered the study area (i.e., field of view) which resulted in higher accuracy.

### 3.3. Performance Evaluation

In order to ensure that the system is more accurate as compared with other previous works, three mathematical equations where implemented such as accuracy (*A*), sensitivity (Sn), and specificity (Sp) as shown in Equations (12), (13), and (14), respectively. There are four main elements integrated in these equations, namely, (i) True Positive (TP) which indicates the number of positive sperm that are correctly recognized by the proposed technique, (ii) True Negative (TN) which indicates the negative sperm samples that are positively recognized by the proposed method, (iii) False Positive (FP) which indicates the number of sperms in which the expert tagged them as negative and the system recognizes them as positive, and (iv) False Negative (FN) which indicates the number of sperm in which the expert tagged them as positive and the proposed algorithm recognizes them as negative.

(12) $$\begin{array}{c} \text{Accuracy }\left(A\right)=\frac{\text{TP}+\text{TN}}{\text{TP}+\text{TN}+\text{FP}+\text{FN}}, \end{array}$$

(13) $$\begin{array}{c} \text{Sensitivity }\left(\text{Sn}\right)=\frac{\text{TP}}{\text{TP}+\text{FN}}, \end{array}$$

(14) $$\begin{array}{c} \text{Specificity }\left(\text{Sp}\right)=\frac{\text{TN}}{\text{TN}+\text{FP}}. \end{array}$$

The article "Multistage Optimization Using a Modified Gaussian Mixture Model in Sperm Motility Tracking" was published in 2021. Journal: Comput Math Methods Med.

## 4. Results

Our results were compared with the other methods such as zero-crossing [33] and classic edge segmentation (Sobel and Prewitt) [34] to evaluate its performance.  Figure 4 shows the comparison results to evaluate the differences between the proposed modified GMM and the other two methods. Classical edge segmentation and zero-crossing techniques included the whole sperm structure (i.e., head, midpiece, and tail) and considered motile and immotile sperms. These approaches add unnecessary noises to the background as compared to our approach. Since the head of the sperm is the brightest part of other sperm's structure as shown in Figure 4(a), our current technique focuses on the head area only to ensure accurate and fast detection. The most important capability that has been noticed in our experiment is that the modified GMM managed to detect all moving object or sperms. Since the main concern in the motility measure is the moving sperms, then, the other undetected sperms are considered immotile.

Moreover, the most important capability of the modified GMM is BG_T_ manipulation. In other words, the background ratio can be modified to get the desired results. The BG_T_ is uniquely assigned based on the sperm video samples. The proposed algorithm able to automatically generate the BG_T_ to ensure robust motile sperm detection.  Figure 5 shows the results of three different background ratios, and for the tested sample, the 50% ratio shows a more accurate, clear image with smooth edges of the moving sperms. However, this percentage is not fixed for all samples.

In terms of the detection accuracy, we also conducted a comparison analysis (performance evaluation) with other techniques such as adaptive threshold which was reported by [35] and global threshold which was reported by [36]. We evaluated 10 different sperm motility video samples whereby each sample consists of different number of sperms. The evaluation is conducted by calculating the accuracy (*A*), sensitivity (Sn), and specificity (Sp) as tabulated in Table 4.

In addition, the overall performance of the proposed method in comparison with the adaptive and global thresholds is presented in Table 5. As we can notice from Table 5, the proposed method attained high accuracy, sensitivity values. Although specificity of the proposed method was not consistent for each sample, this drawback could be improved if the immotile sperms were completely removed from the frame before the tracking process. In addition, observing the quality of the resulted image was not as good as it should be, because the structure of the sperms is still nonuniformed, and some debris and dead cells are still in the foreground as shown in Figure 6. This will affect the analysis and will result in inaccurate results. However, as tabulated in Table 5, in comparison with the adaptive threshold and global threshold, both techniques are still detecting the immotile sperms. This has caused inaccuracy in localizing moving sperms and thus can cause miscalculation in determining sperm velocity. The proposed method can discriminate between moving and nonmoving sperms through an optimization procedure in modified GMM. However, due to the additional optimization steps imposed in the proposed method, the processing time is higher as compared to the two nonoptimized approaches of adaptive and global thresholds.

The article "Multistage Optimization Using a Modified Gaussian Mixture Model in Sperm Motility Tracking" was published in 2021. Journal: Comput Math Methods Med.

Figure 7 shows the error bar for the standard deviation of the results obtained in Table 4 (performance evaluation). As we can see from the graph, our method has the smallest error bar length (specifically the accuracy and the sensitivity) which indicates that these values are concentrated, and the plotted average is more likely as compared to the adaptive and global threshold methods. The standard deviation of specificity of the proposed method is higher as compared to other techniques. This could be due to the 10 sperm samples that we used that have different illumination problems, and thus, each sample has different difficulties in determining a localized area. Apart from that, unlike adaptive and global threshold methods, the accuracy and the sensitivity scored the highest points in our method, and they were not overlapped with other methods; therefore, we can tell that our proposed technique is conclusive.

There are two reasons for this to happen: (1) when the number of the detected objects (i.e., sperms) is relatively small; and (2) when we go back to Equation (14), we can tell that the main variable for this equation is the number of detected TP and TN. For instance, samples 6 to 8 have 50% Sp, that is because the number of detected TP is 1 and the number of detected TN is 1 as well, so that makes the percentage of Sp low which is reflected on the length of its error bar. To solve the aforementioned issues, morphological operation was employed in which the image opening and closing were simultaneously applied to improve the nonuniform sperms. Since there are several structural elements (SE) that can be applied, some SE were examined to find the best SE that can provide a clear and homogenous structure and images.  Figure 8 shows the result of applying different SE to the resulted image frames (from the modified GMM). As we can see from the figure, the results of the morphological images with Line and Cube SE do not provide a uniform sperm's structure as compared with the Disk SE.

The article "Multistage Optimization Using a Modified Gaussian Mixture Model in Sperm Motility Tracking" was published in 2021. Journal: Comput Math Methods Med.

The morphological operation in commonly used sperm detection analysis is reported in [37]. They proposed a method that is based on the morphological structure of the sperm using ellipse detection. In this method, gray color is converted to RGB; then, multiple enhanced filters were added to enhance and segment the sperm from the background. However, in our proposed method, the modified GMM is able to convert image class, segmentation, and edge detection and filter the sperm at the same without adding further instructions. This made our proposed method less complex with faster execution. Additionally, the proposed system will detect motile and immotile sperms which could add further noise in velocity measurements. According to Mahdavi et al. [37], the system detects shapes with an ellipse structure only which is not reliable, because they could be other dead cells or debris in the solution that has an ellipse shape.

Sperms' coordinate in the current, and the previous frames are needed to calculate the velocity of the sperm. The similarity index was proposed in this study with a certain threshold. The results of the tracked coordinates are updated and stored automatically in a matrix once each 10 frames. The results of tracking are shown in Figure 9.

In most cases of the sperm tracking, there will be instances of sperm exiting the frame/field of view or sperm entering the frame as shown in Figure 9. These sperms will be automatically updated and do not intervene with the results of the velocity. The sperm exiting could result from several reasons, namely, (i) the sperm losing its kinetic energy and dies, (ii) error in tacking, (i.e.) the similarly index exceeding the threshold, and (iii) the sperms that ran out of the scope of the field of view during the microscopic recording.  Figure 10 shows one of the cases of the sperm that left the field of view between the 10^th^ and 20^th^ frames.

Additionally, sperm entering the field of view or the frame is another condition that could occur. This is because either the lost sperm in the previous frame has been updated or it gains a less threshold of similarity index.  Figure 11 shows three additional sperms that were added between the 20^th^ and 30^th^ frames.

The article "Multistage Optimization Using a Modified Gaussian Mixture Model in Sperm Motility Tracking" was published in 2021. Journal: Comput Math Methods Med.

Finally, for the sperm motility analysis results, there are ten samples with similar frame rates of 30 frames per second and an average of 800 frames. The number of sperms is different from that of another sample. Table 5 shows the results of motility measurement. The classification of the fast progressive (FP), slow progressive (SP), and immotile sperms was done according to the WHO standard of sperm motility analysis as shown in Table 1. The motility results were expressed in terms of average velocity (*μ*m/s). As it can be noticed from Table 6, some samples had smaller deviations and others had larger standard deviations. This condition is anticipated because the standard range of either FP or SP is quit wide, due to the different number of sperms in each sample. Additionally, in terms of classification, a sample is considered normal if the percentage of the sum of fast progressive (FP) sperm and the slow progressive (SP) sperm exceeds 40% from the total sperm (immotile + FP + SP).

## 5. Discussions

To understand and verify the results obtained from the previous section, trends of sperm's velocity are plotted in Figure 12 where their velocities have been classified into the WHO standards of either fast progressive, slow progressive, or immotile. Each sample represented a different number of sperms, and from the figure, samples 3, 4, 8, and 9 are considered a normal sample since the fast progressive and slow progressive sperms exceed 40% from the total sperms. The proposed system is capable of automatically classifying the sperm samples based on the calculated sperm's velocity. The proposed optimization technique will ensure sperms are accurately identified, and the nonmoving sperms as well as debris are excluded from the analysis. This advantage will provide an improved sperm motility classification which will eventually aid the male infertility diagnosis.

The velocity variations can be justified by many factors. For example, the size of the middle piece of the sperm is critical because it contains mitochondria which provides the energy in forms of adenosine triphosphate (ATP) for the sperm to live and propagate. The larger the size is, the more fuel it has; therefore, it can move faster. There are studies conducted by [38, 39] that proved the higher potential and the size of middle piece of the sperm results in higher sperm's velocity. The same study also concluded that the length of the sperm plays a role in its velocity and that shows a significant linear relationship between the length of the sperm and its swimming velocity.

Moreover, the number of debris and dead cells surrounding the sperms could lower the speed of the sperm. In general, the existence of the debris near or in the area of sperm could result in many collisions between the moving sperm and other debris and dead cells, and that could reduce the sperm's velocity. In addition to that, the high number of debris represents high viscosity thus eventually reducing the sperm's velocity. We can observe this incidence by comparing the results obtained in Tables 6 and 4, sample results (frames) as shown in Figure 13, respectively. Sample 1 contains a lot of debris and accumulated dead cell; thus, the sample will have high density which will reduce the speed of the moving objects. In the contrary, sample 3 and sample 4 have many sperms with a high-speed value. The two samples also had less debris and dead cells around the sperms, and that could explain the reason that they have an overall high number of fast progressive sperms.

The article "Multistage Optimization Using a Modified Gaussian Mixture Model in Sperm Motility Tracking" was published in 2021. Journal: Comput Math Methods Med.

The number of immotile sperms near the moving sperms may also affect the sperm's velocity. Referring to Table 6, we noticed that the ratio between the numbers of immotile sperms and motile sperms is large in sample 1 and that is an indicator for low velocity value results. On the other hand, sample 3 had less immotile sperm which is why it results in a large number of sperms that have high velocity. This is supported by studies done by [30, 40] where they found out that there is a relationship between the number of dead sperms and overall sperm velocity in a solution; the higher the numbers of dead or immotile sperms, the lesser the velocity of moving sperm. The studies also mentioned that the existence of dead or immotile sperms might result in collisions which slowed down the progression of the sperms. Since the classification of the samples depends on the number of the motile and immotile sperm, the more immotile sperms the sample has, the more likely the sample will be abnormal.

## 6. Conclusions

In this paper, a modified GMM algorithm with the capability in optimizing sperm detection process was proposed for multisperm tracking for male infertility diagnosis. The proposed method consists of two stages where the first stage focuses on accurate sperm detection while the second stage comprises sperm tracking and velocity measurement. Motility results were evaluated, and 10 sperm samples were presented, and the performance of the proposed method was compared with other state-of-the-art techniques. When tested on 10 sperm motility videos, the proposed method attained 92.3%, 96.3%, and 72.4% in accuracy, sensitivity, and specificity, respectively. These performance indicators ranked the proposed method as the highest as compared to the other methods. Based on the video samples, 4 tested samples were classified as normal and the other 6 turned to be abnormal. The main limitation with the current work is that when two sperms collide and move together in the same line, the system will consider them as one sperm. This problem could be fixed with optimized feature extraction technique where more features of collide sperms will be considered to update the sperm tracker in the tracking process. In addition, despite utilizing Euclidean distance and similarity measures in computing sperm trajectory analysis, feature histogram and foreground information could be added as an indicator to select optimum region for sperm tracking. This will enable object information to be extracted to improve the accuracy of the proposed system. The current state of the proposed system requires code optimization to improve the computational efficiency especially when dealing with high concentration sample. Furthermore, the research can be continued by considering a mathematical model in estimation sperm motion. The estimation will be able to aid researchers in predicting the location of the corresponding sperms in the next consecutive frames.

The article "Multistage Optimization Using a Modified Gaussian Mixture Model in Sperm Motility Tracking" was published in 2021. Journal: Comput Math Methods Med.

## Figures and Tables

**Figure 1:** Overall process of the proposed method.

**Figure 2:** Pseudocode of modified Gaussian Mixture Model.

**Figure 3:** Optimization of background threshold.

**Figure 4:** Comparison of sperm detection between proposed method and other method in (a) original frame, (b) classical edge segmentation, (c) zero-crossing, and (d) the proposed method.

**Figure 5:** Comparison of different BG ratio size in (a) original frame, (b) segmented with 90% BG ratio, (c) segmented with 50% BG ratio, and (d) segmented with 20% BG ratio.

**Figure 6:** Debris and nonuniform sperm structure that resulted from the proposed method.

**Figure 7:** Comparison of the performance evaluation between the proposed method and the other common techniques of adaptive and global thresholds. The value presented here is in term of average ± standard deviation.

**Figure 8:** Comparison of different SE for image morphology.

**Figure 9:** Results of sperm coordinate tracking.

**Figure 10:** Illustration of sperm leaving the field of view condition.

**Figure 11:** An example of sperm reentering the image frame.

**Figure 12:** Trends of sperm velocity that have been classified for 10 sperm samples.

**Figure 13:** Sperm movement scenario for (a) sample 1, (b) sample 2, (c) sample 3, and (d) sample 4.

**Table 1:** WHO standard for normal sperm characteristics.

Sperm property	WHO standard for normal sperm property
Sperm count	10 million sperms per milliliter.
Sperm morphology	Head: oval in shape, 3–5 *μ*m long and 2-3 *μ*m wide Middle piece: less than 1 *μ*m in width, 5–7.5 long, and must be uniform and visible Tail: 45 *μ*m in length, uniform, and visible
Sperm motility	Fast progressive: velocity more than 25 *μ*m/s Slow progressive: velocity less than 25 *μ*m/s Immotile: velocity is equal to zero

The article "Multistage Optimization Using a Modified Gaussian Mixture Model in Sperm Motility Tracking" was published in 2021. Journal: Comput Math Methods Med.

**Table 2:** Summary of the previous methods in multiple sperm tracking.

Techniques	Advantages	Disadvantages
CASA [28, 29]	(i) Detect the sperm's features	(i) Requires a big sample (ii) Fails in sperm collisions and proximity
JPDAF [20, 21, 22]	(i) Adaptive learning (ii) Works well with sperm collisions	(i) Computational complexity (ii) Slow process termination
HGDT [23]	(i) Combination of object segmentation and tracking (ii) Self-learning capability	(i) Fails in multiple sperm tracking.
CSR-DCF [30]	(i) Implementing of training and testing data for tracking and features extraction (ii) Usage of sperm's features in tracking	(i) Requires large training data (ii) High computational complexity (iii) Difficult to implement
ADT [26, 31]	(i) Fast execution process (ii) Multisperm tracking	(i) Its efficiency decreases in a high dense medium. (ii) It works poorly when many sperms accumulate in a small space
DAT [27]	(i) Easy to implement (ii) Less mathematical complication	(i) Does not predict the dead and newborn sperms (ii) It does not require a testing data (frames)

**Table 3:** Summary of the previous methods in multiple sperm tracking.

Specification	Specification value/range
Microscope	Olympus CX31
Video camera	Mounted microscope camera UEye UI-2210C
Magnification	×400
Video format	.AVI
Video resolution	640x480
Video duration	2-7 minutes
Frame rate	50 frames/sec
Participants	85 male participants aged 18 years or older

**Table 4:** Sperm detection results of proposed method, adaptive thresholding and global thresholding method.

Sample	No. of motile sperms	No. of immotile sperms	Proposed method			Adaptive threshold			Global threshold		
			*A* (%)	Sn (%)	Sp (%)	*A* (%)	Sn (%)	Sp (%)	*A* (%)	Sn (%)	Sp (%)
1	11	51	91.0	90.0	100	81.3	75.0	81.0	40.0	33.3	46.2
2	9	19	98.0	97.0	97.0	77.8	86.4	79.2	41.2	22.2	62.5
3	21	12	91.3	95.0	98.0	84.6	90.5	80.6	25.8	40.0	40.0
4	19	16	95.0	98.3	66.0	67.5	81.0	72.0	25.0	37.5	20.0
5	16	29	94.4	93.0	96.7	73.8	75.0	72.7	28.1	18.2	33.3
6	9	16	90.0	90.0	50.0	65.7	75.0	60.9	50.0	60.0	45.5
7	6	19	91.2	100	50.0	53.8	42.9	60.0	30.8	33.3	30.0
8	10	15	91.7	100	50.0	65.4	58.8	72.2	37.5	50.0	30.2
9	11	12	92.8	100	66.6	65.7	58.8	72.6	52.2	50.0	53.3
10	7	16	87.5	100	50.0	55.2	58.3	52.9	38.9	25.0	50.0

**Table 5:** Comparison of overall performance between proposed method, adaptive threshold, and global threshold.

Criteria	Proposed method	Adaptive threshold	Global threshold
Accuracy (average ± std)	92.3 ± 2.78	69.1 ± 9.76	37.1 ± 9.04
Sensitivity (average ± std)	96.3 ± 3.89	70.2 ± 14.17	37.2 ± 12.72
Specificity (average ± std)	72.4 ± 21.66	70.4 ± 9.02	41.1 ± 12.17
^∗^Processing time (second)	>1 min	<1 min	<0.5 min
Detected sperm features	Head, midpiece, tail	Head, midpiece, tail	Head, midpiece, tail
Immotile sperms	Not detected	Detected	Detected
Advantage	Able to locate only moving sperms due to optimization algorithm in modified GMM	Accurately detect whole sperm body in less than 1 minute	Accurately detect whole sperm body in less than 0.5 min
Disadvantage	Longer processing time	Unnecessary objects such as immotile sperms and debris are considered, thus causing inaccurate tracking	Unnecessary objects such as immotile sperms and debris are considered, thus causing inaccurate tracking

^∗^Processing time is referred to the time required for the method to accurately track the sperms in the consecutive 50 frames. 50 frames were selected for consistency in comparison.

The article "Multistage Optimization Using a Modified Gaussian Mixture Model in Sperm Motility Tracking" was published in 2021. Journal: Comput Math Methods Med.

**Table 6:** Classification of sperm motility results.

Sample	Immotile sperms	Fast progressive sperms			Slow progressive sperms			Classification
		No. of sperms	Average velocity (*μ*m/s)	Standard deviation	No. of sperms	Average velocity (*μ*m/s)	Standard deviation	
1	51	4	34.5	1.3	7	23.2	4.6	Abnormal
2	19	4	49.5	1.2	5	13.6	7.1	Abnormal
3	12	14	36.9	3.9	7	12.8	4.5	Normal
4	16	10	36.6	4.5	9	4.5	3.05	Normal
5	29	4	27.5	2	12	6.34	4.22	Abnormal
6	16	3	25.9	0.77	6	5.4	2.3	Abnormal
7	19	3	26.2	0.7	3	17.4	2.62	Abnormal
8	15	4	26.2	0.78	6	8.8	5.4	Normal
9	12	4	29.5	4.5	7	4.1	2.54	Normal
10	16	5	27.5	2	2	3.85	1.48	Abnormal

## Data Availability

The VISEM Multimodal video dataset of human spermatozoa used to support the findings of this study have been deposited in the name of VISEM repository https://datasets.simula.no/visem/.
